This article has been retracted.

# Unleashing the horizons of labor quality, digitalization on upgradation of industrial structure in Asian economies

**DOI:** 10.1371/journal.pone.0288866

**Published:** 2023-07-18

**Authors:** Zujie Zhang, Ghulam Rasool Madni, Jaweriya Naeem

**Affiliations:** 1 School of Economics and Management, Beijing Jiaotong University, Beijing, China; 2 Division of Management and Administrative Science, Department of Economics, University of Education, Lahore, Pakistan; 3 Department of Economics, University of Education, Lahore, Pakistan; Xuzhou University of Technology, CHINA

## Abstract

A country’s industrial structure plays a pivotal role in determining its competitiveness, growth, and sustainability. Recently, many Asian countries have experienced significant economic upgradation and transformation and have emerged as major players in global trade. It is crucial to understand the factors contributing in upgradation of industrial structure of Asian economies for their continuous progress and it is little focused in literature. This study explores the effect of labor quality and digitalization on the upgradation of the industrial structure in 32 Asian countries covering the time period from 2010–2021. Multiple econometric techniques are applied for a comprehensive analysis of data, and the findings show that high-quality labor has a positive contribution to upgrading the industrial structure. Moreover, digitalization upgrades the industrial structure by improving connectivity, fostering collaboration, and enhancing productivity. Based on the findings of this study, Asian countries should prioritize investments in education and skill development to enhance human capital quality. Additionally, they should promote policies that facilitate digitalization, including investments in digital infrastructure, the development of digital skills, and the creation of a supportive regulatory environment. Thus, Asian countries can accelerate the upgradation of their industrial structure, leading to sustainable economic growth, increased competitiveness, and improved living standards.

## 1. Introduction

The term "upgradation of industrial structure" is a process of improving or advancing existing industrial infrastructure within a given sector or region [1]. It involves modernizing and enhancing various aspects of industrial operations, such as technology, processes, equipment, and overall efficiency, to drive economic growth and competitiveness [2]. The upgradation of industrial structure can encompass several dimensions, including technological advancement, infrastructure development, skills development, and research and development [3–5]. How developing economies can upgrade their industrial structures is a matter of great concern. It is yet unknown how technological advancement and labor quality affect industrial upgradation [6] because the effects of labor quality and technology are rarely supported by empirical evidences [7, 8].

Industrial upgradation and technological advancement (digitalization) are closely interconnected. Technological advancement plays a significant role in upgradation of industrial structures, whereas industrial upgradation, in turn, fosters and encourages further technological innovation [9]. The impact of technological advancement on upgradation of industrial structure can be observed through many channels, such as automation, advanced machinery, process optimization, innovations, and environmental sustainability [10]. Automation and advanced machinery enable faster and more accurate production processes and enhance the overall operational performance [11]. Industries can achieve higher output levels with fewer resources, leading to increased productivity [12]. Advanced technologies offer opportunities for process optimization within the industrial sector [13]. With the help of advanced technology, industries can identify inefficiencies and areas of improvement. Technological advancement fosters innovation within industries, leading to the development of new products, services, and business models [14–16]. Modern technologies enable industries to gather insights, identify market trends, and respond quickly to changing customer demands through the introduction of new and improved products, along with the exploration of new markets [17–19]. Adopting advanced technology is essential for industries to remain competitive in the global market. Industries that successfully leverage technology to upgrade their structures have a competitive edge. They can offer innovative products, improve customer experiences, and optimize supply chains. This enhances their ability to compete in domestic and international business landscapes [20]. The technological advancement is usually proxied by digitalization. Digitalization is the process of integrating data-driven processes and digital technologies into numerous facets of industrial operations [21]. Industries can modernize their industrial processes using digital technologies to streamline operations and maximize resource use [22]. The improvement of industrial structure is accelerated by this connectedness, which encourages collaboration, supply chain optimization, and innovation [23]. Digitalization has a role in upgradation of industrial structure by enabling automation, data-driven decision making, enhanced connectivity, flexibility, improved customer experiences, and fostering innovation [24]. Embracing digital technologies and integrating them into industrial operations is key to staying competitive, driving growth, and achieving sustainable development in the evolving digital era [25].

The relation between labor quality and upgradation of industrial structure is interdependent. Labor quality refers to the skills, education, and capabilities of labor [21]. The labor quality impacts the upgradation of industrial structure in many ways as upgrading industrial structure often involves the integration of advanced technologies and automation [22]. A skilled and adaptable workforce is crucial for effectively utilizing and managing these technologies [23]. Highly skilled workers can quickly adapt to new technologies, operate complex machinery, and maximize productivity [24]. Labor quality plays a vital role in driving innovation and research within industries. Skilled workers with expertise in research and development (R&D) contribute for development of new technologies, products, and processes [25]. Their knowledge and creativity fuel the upgradation of industrial structure by introducing cutting-edge solutions and advancements [26]. Skilled labor tends to be more productive and efficient. Workers with specialized skills and training can perform tasks more accurately, quickly, and with fewer errors [27]. A well-trained and adaptable workforce can quickly learn new techniques, work with advanced equipment, and embrace new methodologies [9]. Skilled workers are crucial for maintaining quality control and assurance standards during the upgradation of industrial structure [28]. They possess the knowledge and expertise to identify and rectify issues, implement quality management systems, and ensure that upgraded processes meet industry standards [29]. Investing in the development of a skilled workforce is crucial for successful and sustainable upgradation efforts, enabling industries to stay competitive in a rapidly changing economic landscape [30, 31].

This paper discusses the importance of upgradation of industrial structure in context of labor quality and digitalization in Asian countries. Most economies in Asia have experienced significant structural change over the past four decades, particularly in the structure of their output and employment systems. The production and export systems of the East Asian economies underwent considerable transformations beginning in the 1960s and 1970s [32–34]. These economies saw considerable economic and industrial upgrading, first in Japan and East Asian countries, then in Southeast Asia, and finally in China [35–38]. The fact that “India’s 2011 National Manufacturing Policy aimed to increase manufacturing’s contribution to the GDP to 25% while creating 100 million manufacturing jobs, speaks about the country’s belief in upgrading the industrial sector” [11]. The Philippines created a thorough manufacturing road map in an effort to reverse over 50 years of steady deindustrialization [39]. In 2014, Indonesia adopted a new Industry Law. Through its "Made in China 2025" program, China is promoting high-tech sectors and usage of technology in its production sector [40].

Asian economies enjoyed rapid growth over the past decades, and their industrial sectors have played a central role in driving this growth [41]. Understanding the relation between labor quality, digitalization, and industrial upgradation can provide insights into how these countries can sustain and further enhance their economic development. Enhancing labor quality and adopting digital technologies can contribute to higher productivity, innovation, and efficiency, thereby strengthening the industrial structure [42]. A comprehensive understanding of the impact of labor quality and digitalization on industrial upgradation is crucial for promoting inclusive growth [43] and socioeconomic development in Asian countries [44]. This study collected the panel data of 32 Asian countries for the period of 2010–2021 to find the relationship among labor quality, digitalization and upgradation of industrial structure. There are several novel and significant reasons to study the impact of labor quality and digitalization on the upgradation of industrial structure in Asian countries. The earlier literature very little focused on this dimension while Asian countries have experienced rapid economic growth and industrialization in recent decades. Understanding the role of labor quality and digitalization in the upgradation of industrial structures is crucial for sustained growth and enhancing competitiveness in the region. Moreover, Asian countries are characterized by diverse labor markets with varying levels of education, skills, and expertise. Studying the impact of labor quality on industrial upgradation provides insights into how skill development, education systems, and workforce training programs can contribute to enhancing industrial productivity and efficiency. The findings can facilitate the policy decisions, fostering regional collaboration, and contribute to knowledge about the broader implications of labor quality and digitalization in industrial transformation.

### 1.1. Objectives of the study

- To determine the impact of labor quality and digitalization on upgradation of industrial structure in Asian economies
- To examine the mechanisms affecting labor quality and digitalization through mediating factors.
- To suggest policies based on empirical estimations.

The remainder of this paper is organized as follows. Section 2 explains the methodology, data, and the estimation techniques used. Section 3 highlights the empirical results and discussion, and Section 4 concludes the study along with policy recommendations.

## 2. Methodology

### 2.1. Model

Aforementioned debate highlights that digitization and the quality of human capital are both continually improving in Asian nations. The industrial structure is also continually being upgraded at the same time. The general theory of industrial upgradation and human capital states that, to some extent, the cadence and rhythm of industrial upgrading are determined by the quality of human capital [45]. When it comes to attracting in foreign investment and encouraging the adoption of new technologies, human capital quality is crucial. As a result, the following theoretical claim has to be verified: The industrial structure is determined by human capital [46]. The "digital economy" in the broader sense “integrates all digitally oriented economic activities, using the digitization of ICT as a key production factor, using contemporary information and communication infrastructure as a carrier, and offering goods or services with digital components. After the agricultural and industrial economies, the digital economy has emerged as a new economic form in recent years” [47]. The digital economy has become more significant in economic and social activities [48]. The broader premise is that industrial upgrading’s organizational structure is determined by digitalization. As a result, the measurement model in this paper is devised as follows:

$$IDS_{it}=\alpha_{0}+\alpha_{1}HQL_{it}+\alpha_{2}DIG_{it}+\alpha_{3}INF_{it}+\alpha_{4}YPC_{it}+\alpha_{5}FDI_{it}+\alpha_{6}HTX_{it}+u_{i}+v_{it}+\varepsilon_{it}$$ (1)

In Eq (1), IDS represents the industrial structure of an economy *i* in time *t*. HQL is quality of human capital, DIG shows the digitalization, inflation is INF, per capita GDP is YPC, foreign direct investment is FDI, and HTX show export of high tech products. *u*_*i*_ is an “individual fixed effect”; *v*_*t*_ is a “time fixed effect”; *ϵit* is a “random error term”.

This research also examined the affecting mechanism of quality of human capital and digitalization on upgradation of industrial structure of Asian countries through three mediating factors: institutional quality, unemployment rate and research and development expenditures by government. Among those, Eqs 2 and 3 show the mediating effect of institutional quality, Eqs 4 and 5 represent the mediating effect of unemployment while Eqs 6 and 7 show the mediating effect of research and development expenditures.


$$ISQ_{t}=\alpha_{0}+\alpha_{1}HQL_{it}+\alpha_{2}DIG_{it}+\alpha_{3}INF_{it}+\alpha_{4}YPC_{it}+\alpha_{5}FDI_{it}+\alpha_{6}HTX_{it}+u_{i}+v_{it}+\varepsilon_{it}$$ (2)

$$IDS_{t}=\alpha_{0}+\alpha_{1}HQT_{it}+\alpha_{2}HQL_{it}+\alpha_{3}DIG_{it}+\alpha_{4}YPC_{it}+\alpha_{5}FDI_{it}+\alpha_{6}HTX_{it}+\alpha_{7}ISQ_{it}+u_{i}+v_{it}+\varepsilon_{it}$$ (3)

$$UEM_{t}=\alpha_{0}+\alpha_{1}HQT_{it}+\alpha_{2}DIG_{it}+\alpha_{3}INF_{it}+\alpha_{4}YPC_{it}+\alpha_{5}FDI_{it}+\alpha_{6}HTX_{it}+u_{i}+v_{it}+\varepsilon_{it}$$ (4)

$$IDS_{t}=\alpha_{0}+\alpha_{1}HQT_{it}+\alpha_{2}HQL_{it}+\alpha_{3}DIG_{it}+\alpha_{4}YPC_{it}+\alpha_{5}FDI_{it}+\alpha_{6}HTX_{it}+\alpha_{7}UEM_{it}+u_{i}+v_{it}+\varepsilon_{it}$$ (5)

$$RAD_{t}=\alpha_{0}+\alpha_{1}HQT_{it}+\alpha_{2}DIG_{it}+\alpha_{3}INF_{it}+\alpha_{4}YPC_{it}+\alpha_{5}FDI_{it}+\alpha_{6}HTX_{it}+u_{i}+v_{it}+\varepsilon_{it}$$ (6)

$$IDS_{t}=\alpha_{0}+\alpha_{1}HQT_{it}+\alpha_{2}DIG_{it}+\alpha_{3}INF_{it}+\alpha_{4}YPC_{it}+\alpha_{5}FDI_{it}+\alpha_{6}HTX_{it}+\alpha_{7}RAD_{it}+u_{i}+v_{it}+\varepsilon_{it}$$ (7)

The details of the variables are as following:

Industrial Structural Upgradation: This paper fundamentally observes the potential determinants affecting the upgradation of industrial structure in Asian countries. Industrial structural upgradation is measured as “weighted sum of industrial structural indicators”. The calculation formula is *Y = Σ*_i_*Z_*i*_ = 1*Z_*1*_+2*Z_*2*_+3*Z_*3*_ where *Y* is “an index of industrial structural upgradation” and *Z*_*i*_ represents “proportion of the output value of the *i*^*th*^ industry to the total output value”. The value of *Y* near to 1 represents that there is slow upgradation of industrial structure while value of Y near to 3 shows the fast upgradation of industrial structure.

### 2.2. Data and sample

To find the impact of digitalization on the industrial structural upgradation, a comprehensive evaluation index system is built. Referring to the studies [36, 44, 49–54], three factors are considered for construction of the index: “digital economy infrastructure”, “digital economy openness”, and “digital technology innovation environment and competitiveness”. The weights and scores of digitalization are calculated through principal component and factor analysis.

The high school enrollment ration is used to gauge the labor quality gained from United Nations Development Program. Export of high-tech products is the proportion of total exports and inflation shows the annual consumer price index. The data of institutional quality is obtained from world governance indicators while research and development is considered as a percentage of government expenditures and employment shows the employment rate in a country. The data is gained from the World Bank, world governance indicators and CEIC. This study selected 32 Asian countries as shown in Table 1 from the perspective of availability of data for the period of 2010–2022.

**Table 1:** Sample countries.

*Armenia*	*Egypt*	*Laos*	*Singapore*
*Azerbaijan*	*India*	*Malaysia*	*Sri Lanka*
*Bahrain*	*Indonesia*	*Maldives*	*Taiwan*
*Bangladesh*	*Islamic Republic of Iran*	*Nepal*	*Thailand*
*Bhutan*	*Iraq*	*Islamic Republic of Pakistan*	*Turkey*
*Brunei*	*Israel*	*Philippines*	*United Arab Emirates*
*China*	*Jordan*	*Russia*	*Uzbekistan*
*Cyprus*	*Kazakhstan*	*Saudi Arabia*	*Vietnam*

When dealing with panel data, choosing the right regression model is essential. Pooled regression, fixed effects, and random effects regression models are typically considered for analysis of panel data. First, the selected model is validated using a pooled regression model. The findings show that regression coefficients are not significant, and the F-test findings at a 1% significance level disprove the original premise that using a pooled regression model would be beneficial. The best estimation strategy is then determined using the Hausman test. As a result, the estimation outcomes obtained through the development of a fixed effect model are regarded as ideal and reliable. It is crucial to keep in mind that using ordinary linear least squares estimation (OLLS) can cause endogeneity problems and result in biased coefficient estimations. Two different estimate techniques, “two stage least squares” (2SLS) and “generalized method of moments” (GMM), have been used to resolve the statistical issues resulting from reverse causality and omitted variables [40, 55].

## 3. Estimated results and discussion

Table 2 displays that the independent variables of quality of human capital quality and digitalization significantly contributes to enhance the industrial structure in Asian countries. The OLS estimation results are shown in columns (1) and (2). In column (1), the findings reveal a positive regression coefficient for human capital quality and digital economy at a 1% significance level, even without considering control variables. This suggests that a unit increase in digitalization and quality of human capital will enhance the industrial structure by 0.27 and 0.135 units, respectively. These results emphasize on significant role played by digitalization, as well as the quality of human capital in improving the industrial structure. Moving on to column (2), the findings reveal that coefficient of digitalization is 0.026 after controlling the factors like capital, inflation, high tech exports, FDI, and per capita GDP. This suggests that the industrial structure will improve by 0.026 and 0.211 units for every unit increase in the development of the digital economy and quality of human capital, respectively. These results add more evidence to the idea that improvement of the industrial structure is significantly influenced by digitalization and quality of human capital.

**Table 2:** Estimated results.

*Variable*	*1*	*2*	*3*	*4*
*IDS*_*t-1*_				*0*.386*** (0.*238)*
*DIG*	*0*.027*** (0.*173)*	*0*.026*** (0.*129)*	*0*.119*** (0.*216)*	*0*.175*** (0.*196)*
*HQL*	*0*.135*** (0.*015)*	*0*.211** (0.*213)*	*0*.198** (0.*258)*	*0*.153*** (0.*253)*
*INF*		*-0*.082* (0.*167)*	*-0*.155** (0.*243)*	*-0*.*095* *(0*.*183)*
*HTX*		*0*.253** (0.*528)*	*0*.416*** (0.*628)*	*0*.367** (0.*571)*
*FDI*		*0*.183** (0.*292)*	*0*.256*** (0.*364)*	*0*.*217* *(0*.*364)*
*YPC*		*0*.083*** (0.*167)*	*0*.193** (0.*364)*	*0*.138* (0.*263)*
*Constant*	*5*.623*** (0.*639)*	*4*.692*** (1.*358)*	*4*.961*** (2.*381)*	
*R* ^*2*^	*0*.*55*	*0*.*65*	*0*.*61*	
*AR (2)*				*0*.*431*
*Hansen Test*			*0*.*673*	

“Robust standard errors in parentheses, AR(2) and Hansen test report the p-value

***p < *0*.*01*

**p < *0*.*05*

*p < *0*.*1*.*”*

Columns (3) and (4) show the outcomes of the 2SLSL and dynamic differential GMM, respectively. It is found that industrial structure of the sample countries improves by 0.119 and 0.198 units, for every unit rise in the level of digitalization and the quality of human capital respectively, showing that the estimation results are still reliable.

Then, the impact mechanism of quality of human capital and digitalization on the upgradation of Asian countries is investigated by building mediating effects models and findings are shown in Table 3. Columns (1) and (2) highlight the findings of institutional quality. These columns show that the digitalization and quality of human capital can significantly upgrade industrial structure in presence of quality institutions and quality of institutions have the capability to improve the quality of human capital and digitalization of the Asian economies. We found that the digitalization and quality of human capital can significantly increase the quality of institutions, thus upgrading the industrial structure. The strong potential of the tertiary sector to apply itself to the digital economy can therefore encourage the upgradation of industrial structure.

**Table 3:** Mediating effects.

	*ISQ*	*IDS*	*UEM*	*IDS*	*RAD*	*IDS*
*DIG*	*0*.051*** (0.*082)*	*0*.042*** (0.*059)*	*-0*.316** (0.*259)*	*0*.253*** (0.*151)*	*0*.398** (0.*428)*	*0*.035*** (0.*128)*
*HQL*	*0*.0136** (0.*052)*	*0*.128*** (0.*165)*	*-0*.463*** (0.*216)*	*0*.0226** (0.*261)*	*0*.528*** (0.*638)*	*0*.361** (0.*231)*
*INF*	*0*.011* (0.*021)*	*-0*.158** (0.*169)*	*-0*.192*** (0.*238)*	*-0*.326** (0.*218)*	*-0*.421* (0.*521)*	*-0*.281* (0.*326)*
*HTX*	*0*.152** (0.*129)*	*0*.238*** (0.*367)*	*0*.234* (0.*258)*	*0*.367*** (0.*236)*	*0*.516** (0.*631)*	*0*.*281* *(0*.*532)*
*FDI*	*0*.163*** (0.*256)*	*0*.152** (0.*364)*	*0*.153** (0.*806)*	*0*.371** (0.*328)*	*0*.118* (0.*281)*	*0*.183* (0.*187)*
*YPC*	*0*.284*** (0.*367)*	*0*.253** (0.*153)*	*0*.311* (0.*316)*	*0*.235* (0.*436)*	*0*.238** (0.*369)*	*0*.286* (0.*367)*
*ISQ*		*0*.248*** (0.*365)*				
*UEM*				*-0*.365*** (0.*215)*		
*RAD*						*0*.528** (0.*341)*
*Constant*	*4*.381** (3.*612)*	*7*.69** (2.*69)*	*5*.39** (3.*617)*	*8*.215** (5.*231)*	*3*.619*** (4.*592)*	*6*.395*** (2.*367)*
*R2*	*0*.*45*	*0*.*61*	*0*.*35*	*0*.*71*	*0*.*63*	*0*.*72*

“Robust standard errors in parentheses

***p < *0*.*01*

**p < *0*.*05*

*p < *0*.*1*.*”*

Columns (3) and (4) show mediating impact of total employment, while columns (5) and (6) show the impact of research and development expenditures by government. It is found that increase in digitalization and quality of human capital causes to decrease unemployment rate significantly decreases and increase in expenditures on research and development by government. The digital economy and quality of human can also contribute to improve the industrial structure by reducing the unemployment rate and increasing the research and development expenditures [56, 57]. “The integration of ICT industries with traditional industries can lead to the expansion of economic scale, especially the growth of online consumption, and thus the effect of consumption-oriented jobs is gradually expanding” [53]. Moreover, “digital technology and quality of human capital can also bring about restructuring of employment. Specifically, the development of digital economy can lead to the creation of more non-farm jobs, providing more employment opportunities and even increasing labor returns, which also increases the share of employment in the service industry” [35].

Our results are in line with those of the majority of research. For instance, it was discovered that the digital economy tended to expand after 1995 [12] and contributed to improve the industrial structure. Our findings differ from earlier research in magnitude but not direction, which may be a function of geographical heterogeneity. Although digitization can significantly contribute to improving industrial structure, its effects may vary depending on a nation’s degree of development [27]. For instance, Myovella et al. [33] used the GMM estimation approach to examine the connection between industrial growth and digitalization in African and the OECD countries. They discovered that usage of internet improves industrial growth in these countries. However, compared to OECD nations, Sub-Saharan Africa is less affected by the impact because of the region’s poor Internet infrastructure. Additionally, it has been discovered that improving the human capital has a substantial impact on upgradation of industrial structure. The results of this study concur with those of older literature, as well. As demonstrated by Lucas [51], who viewed human capital as a primary determinant of economic growth, education is a key catalyst for both industrial growth and structural adjustment. Petrakis and Stamatakis [52] discovered that primary and secondary education have a greater importance for growth in developing nations. In addition, human capital has a large spillover impact that can raise worker productivity and skill levels [53]. From a specific angle, a country’s capacity to modernize its industrial structure is boosted by the amount of human capital it possesses [54].

It is found that FDI has a positive impact on improvement of industrial structure which can be explained in several ways: FDI brings advanced technologies, expertise, and managerial practices from foreign companies to the host country. This transfer of knowledge and technology enhances the capabilities and productivity of domestic industries. Local companies can pick up best practices, enhance their technology infrastructure, and learn from their overseas rivals [55]. This results in the industrial structure’s general modernization and enhancement. Additionally, FDI encourages competition in the industrial sector of the host nation. When foreign companies enter a market, new market dynamics are introduced that motivate domestic companies to increase productivity and efficiency [56]. The competition encourages creativity, the use of novel techniques, and the improvement of industrial methods. As a result, productivity increases and the economy grows as the industrial structure becomes more effective and competitive. FDI frequently offers initiatives and training programs to grow the local workforce. By offering staff opportunities for specialized training and education, foreign businesses invest in the development of human capital. The local workforce’s skills and knowledge are improved, increasing their capacity to operate in modern industries [57]. A skilled labor force boosts the industrial structure as a result, which enhances the industry as a whole. FDI is essential in helping a host nation’s industrial structure become more diverse. In order to create new sectors and opportunities, foreign corporations may invest in domestically undeveloped or nonexistent industries [48]. This diversification lessens reliance on existing industries and lays the groundwork for long-term economic expansion. Additionally, it helps to reduce the dangers brought on by over-reliance on a single industry, strengthening the economy’s resilience.

It is important to note that coefficient of HTX is positive which shows that high tech exports of Asian countries are contributing for upgradation of industrial structure. High-tech exports contribute significantly to economic growth by generating export revenues and increasing GDP [58]. They often command higher prices and profit margins compared to traditional goods, leading to increased profitability and competitiveness. The focus on high-tech exports encourages countries to invest in research and development, innovation, and advanced manufacturing capabilities. This, in turn, drives the improvement of the industrial structure by fostering the development of high-value-added industries. High-tech exports require cutting-edge technologies and continuous innovation. Industries engaged in high-tech exports invest heavily in research and development to create and improve innovative products and services [59]. This culture of innovation spills over to other sectors, driving technological advancement and upgrading the industrial structure as a whole. The adoption and adaptation of advanced technologies in various industries lead to improved productivity, efficiency, and quality [60]. The production and export of high-tech goods necessitate a highly skilled workforce [52]. The emphasis on high-tech exports drives the development of specialized skills in science and technology. The focus on skill development helps to create a pool of highly educated and skilled workers. The presence of a skilled workforce not only supports the high-tech sector but also spurs the other knowledge-intensive industry, contributing to overall improvement of the industrial structure [38].

The impact of inflation on upgradation of industrial structure is found negative for Asian countries. Inflation can have several negative impacts on the improvement of industrial structure as inflation erodes the purchasing power of consumers and businesses [61–63]. Businesses may be reluctant to invest in long-term initiatives or make strategic decisions when inflation is high and unpredictably fluctuating [64]. When pricing and expenses are uncertain, people may adopt a conservative mindset and make fewer investments in R&D, infrastructure, and capacity expansion. This lack of investment may inhibit the development of the industrial structure and the growth of technology [16]. Inflation can skew market pricing signals, making it challenging for companies to determine the relative worth of different commodities and services. Because of misleading signals, businesses may invest in less productive or efficient industries as a result of price distortions [32]. This inefficient use of resources may stop the industrial structure from changing in a way that reflects actual market demands and efficient resource use. Financial markets may become volatile and unstable as a result of high inflation. In response to inflationary pressures, central banks frequently raise interest rates, which can result in more stringent credit requirements and higher borrowing costs for enterprises [42]. This can impede access to capital for investment and limit the ability of industries to improve their infrastructure, adopt new technologies, and drive innovation [42].

The impact of per capita GDP on upgradation of industrial structure was found positive. Higher per capita GDP provides individuals and businesses with increased income, investment capacity, and access to advanced technologies [33, 45]. This, in turn, facilitates the upgradation of industrial structure through increased consumption, investment in infrastructure and technology, and economic diversification. Conversely, the upgradation of industrial structure can contribute to higher per capita GDP by driving productivity, innovation, and competitiveness, leading to sustained economic growth and improved living standards [28, 65].

## 4. Conclusions and policy implications

This research study examined the impact of labor quality and digitalization on the upgradation of industrial structure in Asian countries. This study collected the panel data of 32 Asian countries for the period of 2010–2021. The data is analyzed through OLS regression, 2SLS and GMM techniques. The findings of the study provide some valuable insights into the factors driving the upgradation of industrial structure in the region.

Theoretically, quality of human capital significantly upgrades the industrial structure. The study found the positive and significant impact of labor quality on upgradation of industrial structure in Asian countries. These countries exhibit diverse labor markets with varying levels of education, skills, and expertise. Investing in human capital through education, skills training, and workforce development programs play a pivotal role to increase the industrial productivity and efficiency. Enhancing labor quality through these measures contributes to the upgradation of industrial structure, fostering economic growth and attracting investment.

Moreover, the digitalization has a significant and positive effect on upgradation of industrial structure in Asian countries. It can stimulate the upgradation of industrial structure through strong institutions, total employment and research and development. Digitalization and technological advancement like automation, artificial intelligence, and data analysis have reshaped the industrial operation in Asian economies. Digitalization improve productivity, efficiency, and innovation to enhance the competitiveness of industry in the global market. Adoption of digitalization has become key factor in sustaining growth and driving industrial development.

The findings of the study have important policy implications. Governments in the Asian countries need to recognize the vital role of labor quality and digitalization in upgradation of industrial structure. Policies should focus on investing in education, skills training, and digital infrastructure to nurture a skilled labor force and creation of an environment to enable the technological innovations in the region. This can spur industrial growth, enhancing global competitiveness, and supporting sustainable development in these countries. Moreover, the Asian countries may adopt policies like further opening up their economies and fully utilizing the benefits of labor factors in order to continual upgrading of the industrial structure. The government should actively support its economic development as well as adjustment and optimization of its industrial structure, according to Lin’s theory of "new structural economics" [62]. Additionally, knowledge sharing and collaboration among countries can facilitate the transfer of skills, technology, and expertise, enabling mutual learning and fostering regional industrial integration.

For the purpose of creating successful development strategies and paths, each Asian country should evaluate its advantages and disadvantages in light of digitalization. In order to help the countries having less advanced digital technology in Central and South Asia, the "digital divide" should be bridged by improving the infrastructure in these regions. These nations should prioritize the boosting of specialized talent training, strengthening R&D funding for digital technology, and improving the innovation environment.

In conclusion, this study demonstrates that labor quality and digitalization are pivotal factors in the upgradation of industrial structure in Asian countries. Investing in human capital development and embracing digitalization and technological advancements can lead to increased productivity, efficiency, innovation, and global competitiveness. These findings provide insights that can inform policymakers, industry stakeholders, and researchers in their efforts to promote sustainable industrial development and economic growth in the region.

The limitation of this study is the absence of a more thorough examination of associated theoretical mechanisms. Additionally, a detailed examination of particular problems and deliberate action are needed for the realization of issues of the Asian economies. Another area that requires more research is the heterogeneity of the countries and it should be assessed accordingly.
